RETRACTED

# Intraperitoneal injection of PDTC on the NF-kB signaling pathway and osteogenesis indexes of young adult rats with anterior palatal suture expansion model

**DOI:** 10.1371/journal.pone.0243108

**Published:** 2021-07-09

**Authors:** Yafang Li, Yiqiang Qiao, Huanhuan Wang, Zao Wang

**Affiliations:** 1 Stomatology Department, The First Affiliated Hospital of Zhengzhou University, Zhengzhou, Henan, China; 2 Zhengzhou Stomotology Hospital, Zhengzhou, Henan, China; Qingdao University, CHINA

## Abstract

In recent years, many studies have found that mechanical tension can activiate NF-kB signal pathway and NF-kB plays an important role in the process of osteogenesis. However, it is still unclear whether this process exists in the anterior palatal suture expansion. In this paper, we mainly studied the effect of intraperitoneal injection of PDTC on the NF-kB signaling pathway and osteogenesis index of the anterior palatal suture expansion model in young adult rats. The expansion model is grouped and established: 45 male 8-week-old Sprague-Dawley rats were randomly divided into three groups, an expansion only (EO) group, an expansion plus PDTC (PE) group, and a control group. The results revealed that PDTC inhibited the activity of NF-kB signaling pathway and promote one morphogenetic protein 2 (BMP-2), steocalatin (OCN) expression. Compared with the control group, the optical density (OD) value of BMP in the EO group and PE group rats increased significantly from the first day to the seventh day, and the difference was statistically significant (P<0.05). After 6.0Gy irradiation, PDTC administration group could slightly increase the total SOD level in the liver and serum of rats, and reduce the MDA level in the liver and serum, especially the effect of 60mg/kg and 90mg/kg was the most obvious.

## Introduction

Nuclear transfer factor kB (NF-kB) is an important regulator of nuclear cell gene transcription. It can promote transcription by combining the kB points of various genetic factors. DNA binding proteins. The activation of NF-kB may lead to the excessive appearance of Cain in various sites. At present, researches on exogenous intervention to promote the reconstruction of middle tegmental suture focus on growth factors, drugs and physical stimulation.

In recent years, with the in-depth study and extensive use of the method of expanding the jaw, it has been fully proved that the method can effectively open the middle slit of patients at the peak of growth and development. Maintaining the width of the mid-palatal suture after expansion can help stabilize the effect of maxillary expansion. However, the width of the dental arch after the expansion of the maxillary arch has a tendency to shrink, which is mainly due to the lack of newly formed bone at the mid-palatal seam after the expansion and the lack of sufficient time to mineralize, which is not enough to resist the impact of the palatal horizontal plate. The huge squeezing force of the buccal muscle can easily lead to the absorption of the newly formed bone in the palate tissue. Therefore, the amount of new bone formation and the degree of mineralization of the new bone at the mid palate and the recurrence rate after rapid maxillary arch expansion closely related. Therefore, in order to reduce the recurrence rate after arch expansion in clinic, it is urgent to find a way to promote the formation of new bone and the maturation of mineralization.

RETRACTED

During puberty, increased interdigitated sutures in the pal bone increase resistance to rapid maxillary expansion (RME); this reduces its skeletal effect. Grünheid determined a new method for measuring mid-middle seam maturity, that is, mid-middle seam density ratio, which can be used as an effective predictor of RME bone response. Before the 30 patients (12.9±2.1 years old) who received comprehensive orthodontic treatment received treatment, the pal median suture density ratio, age, cervical spine maturity, and mid bone suture maturity stage were evaluated. Cone beam computed tomography measurements were used to determine the proportion of the prescribed expansion achieved in the larger p-hole, nasal cavity and suborbital foramen [1]. Ye explored the effect of lactoferrin (LF) on the resorption of mesial bone in the palate of rats with rapid cleft palate. He was randomly divided into 3-week-old rats. Computed tomography showed that the bone volume/tissue volume ratio and relative bone density of the sutured bone in the LF group were significantly higher than those in the EO group. Histochemical staining showed that the activity of bone-like cells composed of LF and the amount of new bone formation increased significantly, but there was no significant difference in the activity of osteoclasts. Low frequency stimulates the remodeling process of the bone density and the bone volume sutures under tension in the middle palate. However, this enhancement is not due to reduced bone resorption [2]. The rapid maxillary dilator (RME) has been used for cross-bite after orthodontic treatment, and its overall goal is to enlarge the maxilla by separating the mid-palatal suture. Garrec evaluated the differences in cleft palate expansion among teenagers. Histological studies have dismissed the idea that sutures are fused with age. Three-dimensional radiology has improved our understanding of the response of maxillary expansion, but the resolution of three-dimensional radiology still needs to be improved to fully understand the details of the surrounding maxillary response to RME [3]. Rosa analyzed the promotion effect of laser or LED phototherapy on the formation of mesial bone in the palate after the rapid expansion of the maxilla. He conducted Raman spectroscopy and histological analysis of the suture area and submitted the data for statistical analysis (p≤0.05). In the histological analysis of various inflammations, collagen and osteoblasts have higher activities, while osteoclasts have lower activities [4].

RETRACTED

Innovation points of this paper: In this paper, liver cancer cells were inoculated into the armpit of the right forearm of rats, a tumor-bearing rat model was made, and the rats were given PDTC. The effects of weight changes generally observed in transplanted tumors of different groups of tumor-bearing rats were analyzed, and the tumor suppressive effects of each group were analyzed. The regulation of NF-kB in anterior palatal suture osteogenesis was studied. On this basis, immunohistochemical staining was used to observe the changes of NF-kB expression in in anterior palatal suture.

## NF-kB

### NF-kB composition and activation

In most cells, members of the nuclear transcription factor NF-kB family are usually homodimers or heterodimers (the most common P50 / rela heterodimer), which directly bind the inhibitor protein IBB (IkBα, IkBβ) to form a trimer complex. This is in an inert form to the cytoplasm of many different types of cells. IkB is an activity-inhibiting protein with a molecular weight of 60-70kDa. Its inhibition mechanism is to cover the nuclear localization signal (NLS) on NF-kB, thus preventing NF-kB from entering the nucleus. When the binding site of NF-kB is stimulated by various activation factors such as immunity, NF-kB is activated, and the signal can induce the activation of IkB kinase (IkB Ki2nase, IkK), causing the degradation of IkB [5]. The concrete process is: IKK phosphorylates the 32th and 36th serine of the IK. Beta. A protein of the trimer complex, phosphorylated IkBβ. A is formed by ubiquitin at multiple sites, and finally ubiquitinated ii.beta. Is decomposed by the 26S proteosome and exposes nuclear localization. Signal transduction (RLS) of NF protein rapidly shifts the nucleus to the nucleus (KB site) of the target gene and regulates the NF-kB response. There are many factors that can activate NF-kB, including various stress stimuli, ultraviolet radiation, bacterial mucopolysaccharides, viruses, oxygen free radicals, and various cytokines, immune receptors, enzymes, etc., which are activated by different mechanisms. NF-kB is involved in the physiological and pathological processes of the body’s inflammatory response, immune response, oxidative damage and apoptosis. Inhibitors of NF-kB activation include various antioxidants, such as dithiocarbamate pyrrolidine (PDTC), acetylcysteine, etc.; PDTC is a specific inhibitor of NF-kB. Protease inhibitors such as MG-132; glucocorticoid drugs such as prednisone, dexamethasone. and salicylate preparations such as aspirin [6].

RETRACTED

Metallothionein (MT) is a cysteine-rich metal-binding protein that can remove hydroxyl groups and belongs to the category of antioxidants. It also reverses the activation of NF-kB [7]. When the cells are stimulated, NF-kB can simultaneously control the expression of Ikβa, the mechanism of which is through inducible self-regulatory pathways [8]. Ikβa is a physiological inhibitor of heterodimer NF-kB, and its expression is induced by NF-kB. In human T cells activated by phorbol ester (PMA) or tumor necrosis factor (TNF-α), this particular inhibitor is also degraded as NF-kB is released and enters the nucleus, after which NF-kB is reversely induced Ikβa protein synthesis [9]. There is a negative correlation between SOD activity and MDA concentration [10].

### NF-kB signal system

Including NF-kB/Rel protein family, NF-kB inhibitor protein (inhibitor of NF-kB, IkB) family and IkB kinase (IkB Kinase, IKK). The NF-kB/Rel protein family in the mammals includes NF-kB1 (p50), NF-kB2, (p52), RelA (p65), RelB and C-RelS members, so it is called NF-KB/Rel In the family, the amino terminus contains a conserved Rel homology domain (Rel Homology Domain, RHD) consisting of about 300 amino acids [11]. Usually in the Rel homology region (RHD) of NF-kB, the two Ig-like folded configurations are connected to each other by means of flexible linker segments to form homo- or heterodimers [12]. Dimers with transcriptional activity are P50/c-Rel, PSO/P65, P65/c-Rel and P65/P65, and may also include P50/P50,. P52/P52. The most common activated form of NF-kB, P50/RelA (P50/P65), is a heterodimer [13]. In general, the NF-kB referred to is P50/P65, which is the most widely distributed, the most abundant, and biological. It also has the highest activity and has a central pivotal function in regulating target genes encoding multiple inflammatory factors. The main function of the Rel homology region is to mediate its interaction with family members of the NF-kB inhibitory protein (IkB) [14]; mediate the binding of the Rel protein to specific sequences on DNA; mediate the interaction between the Rel protein and Homologous or heterologous subunits form dimers [15]; they will carry nuclear localization signals and transfer the nuclear factor-rxB involved in activation from the cytoplasm to the nucleus [16]. kB is another protein family in the cytoplasm, and is an inhibitory factor [17]. The main role is to combine with Rel/NF-kB protein in the cytoplasm to form a trimer, so that NF-kB remains in the cytoplasm in an inactive state. The IkB family acts as an inhibitor of intracellular NF-kB [18], and its family members include IkBa, IkBp, IkBy, IkBs, IkB-R, Bcl-3, P100, and P105, of which IkBa and IkBβ dominate. The main functions of IkB protein are: prevent NF-kB from transferring into the nucleus; prevent NF-kB from specifically binding to DNA [19]; Gradually dissociate the NF-KB DNA complex. The IKK complex is composed of three subunits a, β and γ, all of which have similar structural characteristics and high homology [20]. IKKα and IKKβ play an important role in the phosphorylation of IxB specific sites. When IKKα is degraded in the cytoplasm, P50/P65 activates into the nucleus and binds to the KB site of 1KKα [21], which rapidly induces the transcription of IKKα mRNA and protein synthesis. The newly synthesized IKKα enters the nucleus, induces the dissociation of P50/P65 from DNA, and transports P50/P65 back to the cytoplasm to be reused, indicating that P50/P65 and kB constitute a feedback regulation system [22].

RETRACTED

In the resting state, they are combined with their inhibitory subunit of NF-kB (IkB) in the form of dimer and exist in the cytoplasm. When cells are exogenously stimulated, NF-kB activates and functions in the nucleus. One of the classical pathways of NF-kB activation is that NF-kB induced kinase is activated by activator, activates IKK, and phosphorylates the ser 19 and ser23 residues of the ikba-n terminal. In case of IKKβ, ser157 and ser161 residues. Phosphorylation of IkB covalently binds to multiple ubiquitin molecules [23]. Ubiquitination of lkba causes structural changes. The ATP dependent 26S proteasome recognizes and decomposes IkBα. NF-kB is activated as a dimer, enters the nucleus and specifically binds to the KB sequence of the target gene. Start or enhance transcription of certain genes. Nf-rb can also be activated through an alternative pathway. Under normal conditions, the TN receptor (TNVR) phosphorylates Ikα through action, binds to the RelB heterodimer in the matrix, and is selectively activated by the NF-kB/P100 precursor protein into the nucleus, thereby promoting Transcription of target cells. Oxidative stress can activate NF-kB through atypical pathways. External stimuli activate one or more signal transduction pathways, increase intracellular reactive oxygen species (ROS), activate tyrosine kinase (TK), and catalyze a variety of protein kinases, IkB is degraded and activates NF-kB to enter the nucleus to play a role.

RETRACTED

### Role of miR-21 in bone remodeling

miRNA is a type of endogenous non-coding RNA molecule with a length of about 22 nucleotides. Mature miRNAs are produced from primary transcripts through a series of nuclease cleavage processes. The most primitive pri-miRNA, after one processing, becomes pre-miRNA, that is, miRNA precursor, pre-miRNA is digested by Dicer enzyme, and becomes mature miRNA, which is then assembled into RNA-induced silencing complex, which is passed through alkali recognize the 3’non-coding region of the target mRNA by complementary pairing, and guide the silencing complex to degrade the target mRNA or suppress the translation of the target mRNA according to the degree of complementarity, and regulate gene expression at the post-transcriptional level. Current research shows that miRNA has been widely involved in a series of important processes in life, including cell proliferation and differentiation, biological development, disease occurrence, and development. It is speculated that about 60% of the coding genes in the human genome are regulated by miRNA. More and more studies have shown that miRNA is closely related to bone formation. For example, miRNA-214 directly regulates target gene ATF4 to inhibit osteoblast osteogenesis; miRNA-4739 inhibits the expression of target gene LRP3, thereby inhibiting some signaling pathways related to osteogenic differentiation, such as TGF-β pathway and MAPK pathway In turn, it inhibits the osteogenic differentiation of bone marrow mesenchymal stem cells. miR-21 is the first miRNA molecule discovered and confirmed in mammals. Currently, miR-21 has been found in various tissues and cells in 31 species, but it has not been found in plants. miR-21 plays an important role in the occurrence and development of various tumors and cardiovascular diseases. In addition, many in vivo and in vitro experiments have shown that miR-21 is closely related to the osteogenic differentiation of stem cells. For example, miR-21 and BMP9 can synergistically activate the BMP9/Smad signaling pathway and promote the osteogenic differentiation of murine multidirectional differentiated cells; miR-21 can also promote the osteogenic direction of human mesenchymal cells by inhibiting the expression of SPRY2.

The expression level of miR-21 in periodontal ligament stem cells under mechanical stimulation increased, and it was significantly different from that in periodontal ligament cells without stress. According to bioinformatics predictions, the target genes of miR-21 are significantly enriched in signaling pathways related to osteogenic differentiation, such as Jak-STAT signaling pathway and MAPK signaling pathway. miRNA-21 can promote osteogenic differentiation of periodontal ligament stem cells by acting on activin receptor 2B. However, the effect of miRNA-21 on the bone reconstruction of the anterior palatal suture caused by the effect of expansion is not clear.

RETRACTED

## Experimental design of an expanded model of anterior palatal suture in adult rats

### Experimental animals

Healthy SPF-class young adult rats were provided by the SPA Animal Experiment Center of a medical university and given conventional feed (protein 20%-50%, fat 5%.10%, crude fiber 3%.5%).

All rats were euthanized in a CO_2_ gas chamber. The animal studies were approved by the Animal Ethics Committees of Zhengzhou University. Animals were housed and treated under the approved protocols. All rat work was consistent with the requirement of the Animal Ethics Committees of Zhengzhou University. (No. 2018092B).

### Experimental design

Prepare RPMI-1640 medium containing 10% fetal bovine serum, 100 μl/m penicillin and 100 μl/m streptomycin, pu liver cancer cells into it for cultivation, and then incubate at 37°C, 5% CO_2_ to cultivate. The cells grow adherently. After being covered with the whole culture flask, they are passaged with 0.25% trypsin digestion and passaged once every 2–3 days. The exponential growth phase cells were prepared into a cell suspension with a concentration of 1.0x10^7^/ml (the cell viability was determined to be above 95% by trypan blue) for use.

45 male 8-week-old Sprague-Dawley rats were randomly divided into three groups, an expansion only (EO) group, an expansion plus PDTC (PE) group, and a control group. 15 rats in each group were randomly divided into 3 groups by different expansion periods: 1, 4, 7 days. All animals were fed with powder food. A cell suspension containing tumor cells with a concentration of l×l0^7^ cells/ml was prepared, and rats in each group were subcutaneously inoculated with the right forelimb axillary. Each rat was inoculated with 0.2 ml of cell suspension and fed daily to observe the tumor growth of the rats. One week after inoculation, each group of rats can palpate the tumor (the body of the tumor is larger than 1mm×1mm), observe the quality of life of the rats in each group within 50 days, measure the weight every 10 days, and observe the cell volume with a microscope. The second batch is used for radiation experiments.

Immediately after blood sampling, the rats were sacrificed by cervical dislocation and fixed on anatomical plates. After iodine disinfection, the abdominal cavity was opened along the midline of the abdomen, and two pieces of central liver tissue were taken. A piece is trimmed to a size of about 1cm×0.5cm×0.3cm, placed in a ampule containing 4% paraformaldehyde in advance, fixed for 12 hours, and sent to a hospital pathology department for routine dehydration, transparency, and embedding into a tissue wax block for preservation. Complete paraffin section and routine HE staining. The other piece weighs about 1.5 grams. Remove the connective tissue as much as possible and place it in a Petri dish placed on ice. Rinse twice with PBS, cut with ophthalmic scissors, and add 0.25% pancreatin at a rate of 3 ml pancreatin per gram of liver tissue. After that, put the culture dish in a 37°C incubator for 30 minutes for digestion, remove the culture dish, add 10% calf serum at a rate of 3 ml per gram of liver tissue to terminate the digestion, and then pour the digested cell suspension into the pad Filter the glass funnel with 4 layers of gauze into a 15 ml centrifuge tube, centrifuge at 1000 rpm at 4°C for 10 minutes, discard the supernatant, add 5ml of PBS, place the centrifuge tube on a vortex suspension, and dissolve the precipitated cells by shaking For the cell suspension, mix 100 μl of the cell suspension with 100 μl of 0.4% fetal blue solution and inject it into a cell counting plate. After counting the cells under a microscope, dilute the cell suspension with PBS to 1.0×10^7^ cells/ml; Take 1 ml of the above diluted cell suspension into a 1.5 ml EP tube, centrifuge at 1000 rpm for 10 minutes, and discard the supernatant to obtain pelleted cells.

RETRACTED

The positive reaction product of NF-kB P65 is distributed in the cell cytoplasm and (or) cell nucleus and is yellow or brownish yellow. Blue stained cells are negative cells stained with hematoxylin. Comprehensively consider the percentage of stained cells and the degree of staining for evaluation and analysis, semi-quantitative judgment results, randomly select 5 high-power field (x20) tumor tissue areas per slice, and divide them into 4 levels according to the proportion of positive cells in the observed cells: The number of positive cells is less than 10/high power field is negative (-); the number of positive cells is 10–29 cells/high power field is weak positive (+); the number of positive cells is 30-99/high power field is moderately positive (++); The number of positive cells ≥100/high power field is strong positive (+++). In the process of statistical analysis, weak positive, moderate positive and strong positive are treated as positive results.

### Statistical methods

Statistical analysis was performed using SPSS 17 software. Immunohistochemical staining analysis is to use X^2^ test to analyze the correlation between the immunohistochemical results and clinical pathology of NF-kB P65, and the expression in liver cancer lesions after treatment. Taking a = 0.05 as the test standard, it has statistical significance when P<0.05.

RETRACTED

### Ethics statement

All rats were euthanized in a CO_2_ gas chamber. The animal studies were approved by the Animal Ethics Committees of Zhengzhou University. Animals were housed and treated under the approved protocols. All rat work was consistent with the requirement of the Animal Ethics Committees of Zhengzhou University. (No. 2018092B)

## Experimental analysis of the anterior palatal suture expansion model

### Analysis of the effect of PDTC on body indexes of adult rats

As shown in Table 1, Table 2 and Fig 1. PDTC intervention significantly increased the expression of PGC-1αmRNA and PGC-1βmRNA (P<0.01) expression, enhance the formation of intracellular mitochondria in extensor digitorum longus muscle of high-fat rats, and endurance exercise and PDTC had an interactive effect on the expression of COX4 gene in extensor digitorum longus muscle of high-fat rats. Further analysis showed that endurance exercise can increase COX4 mRNA expression in extensor digitorum longus muscle of high-fat rats (P<0.05), while PDTC can weaken endurance exercise to increase COX4 gene expression (P<0.05). Endurance exercise and PDTC intervention have an interactive effect on the expression of PDK4 mRNA in soleus muscle of high-fat rats, and the two synergistically promote the increase of PDK4 expression.

**Fig 1:** Effect of PDTC on relative gene content of rats in extensor digitorum longus muscle of rats.

**Table 1:** Effect of PDTC on the relative content of various genes in the extensor digitorum longus.

	H	HE	Exer	PDTC	E*P
PGC-1a	1	0.63	F = 0.84	F = 18.05	F = 1.72
PGC-1β	1	0.57	F = 0.61	F = 0.00	F = 0.07

H = high-fat rat extensor digitorum longus muscle, HE = high-fat rat extensor digitorum longus muscle COX4 gene expression, Exer = high-fat rat extensor digitorum longus muscle COX4 mRNA expression, E*P = high-fat rat soleus muscle PDK4mRNA expression.Data represents the relative content of SPSS statistics.

**Table 2:** Effect of PDTC on the relative content of various genes in soleus muscle of rats.

	H	HE	Exer	PDTC	E*P
PGC-1a	1	0.93	F = 0.05	F = 0.02	F = 0.00
PGC-1β	1	0.43	F = 0.54	F = 0.12	F = 1.37

H = high-fat rat extensor digitorum longus muscle, HE = high-fat rat extensor digitorum longus muscle COX4 gene expression, Exer = high-fat rat extensor digitorum longus muscle COX4 mRNA expression, E*P = high-fat rat soleus muscle PDK4mRNA expression.Data represents the relative content of SPSS statistics.

### OD analysis of osteogenesis index

As shown in Fig 2, in order to clarify the impact of PDTC intervention on the osteogenic index responsiveness of young adult rats, we detected the OD value of BMP-2 and OCN. Compared with the control group, the OD value of BMP in the EO group and PE group rats increased significantly from the first day to the seventh day, and the difference was statistically significant (P<0.05). When comparing the rats in the EO group and the PE group, it was found that the OD value of BMP-2 in PE group was higher than that of the EO group, and the difference is statistically significant.

RETRACTED

**Fig 2:** OD value of BMP-2、OCN in young adult rats with anterior palatal suture expansion model and PDTC intervention. A: BMP-2; B:OCN; *Statistically significant increase versus the control group (*p < 0.05, **p < 0.01); EO: expansion only group; PE: expansion plus PDTC group.

As shown in Fig 3, during the experiment, rats with stable vital signs, no mucosal infection or other diseases, and no expansion of the expander were included in the statistical scope for tissue sectioning and staining. The weight of the rats in each group was tested. As shown in Fig 3, it was found that the weight of the rats in the non-expanded group showed a steadily increasing trend, while the weight of the rats in the expanded group decreased significantly in the first 3 days after the placement of the helix springs. From the 4th day, the body weight of the rats began to increase gradually. This phenomenon is mainly due to the discomfort of the rats in the expanded group when they first were placed the helix springs, which will affect their normal eating, resulting in a significant trend of weight loss in the first 3 days after the springs is placed: Gradually adapt to the appliance, so from the 4th day, food intake tended to be normal, and the weight increased steadily. Throughout the experiment, the weight of the rats in the expanded group was smaller than that in the non-expanded group (P<0.05), but there was no significant difference in the weight of the rats in the unexpanded group and the expanded group group (P>0.05). The relationship between miR-21 and osteogenesis is shown in Fig 4.

**Fig 3:** Changes in body weight of four groups of rats over time during the experiment.

**Fig 4:** miR-21 is related to osteogenesis.

### Analysis of the protective effect of PDTC on oxidative damage in rats

The body generates oxygen free radicals through enzyme systems and non-enzyme systems, which can attack unsaturated polyunsaturated fatty acids (PUFA) in biofilms, trigger lipid peroxidation, and thus form lipid peroxides. Such as aldehyde groups (malondialdehyde MDA), ketone groups, hydroxyl groups, carbonyl groups, hydroperoxy or internal peroxy groups, and new oxygen radicals. Lipid peroxidation not only converts active oxygen into active chemical agents, that is, non-free radical lipid decomposition products, but also amplifies the role of active oxygen through chain or chain branch reactions. Therefore, an initial active oxygen can lead to the formation of many lipid decomposition products, some of these decomposition products are harmful, and others can cause cell metabolism and dysfunction, and even death. Oxygen free radicals not only cause cell damage through the peroxidation of PUFA in the biofilm, but also cause cell damage through the decomposition products of lipid hydroperoxides. Therefore, the amount of MDA tested can often reflect the degree of lipid peroxidation in the body, and indirectly, the degree of cell damage.

RETRACTED

As shown in Figs 5 and 6, after the body receives ionizing radiation, it will interfere with the body’s antioxidant defense system, destroy the redox balance in the cell, and cause damage to the body. This damage is mainly related to excessive free radicals produced by the body. Proteins are the main targets of free radicals and other oxidants. It is estimated that free radicals scavenged by proteins account for 50% to 75% of the total active free radicals in the macromolecules in the cell. Since certain proteins have a long half-life, it is easy to cause the accumulation of oxidative damage, so the formation of protein oxidative damage may be a highly sensitive indicator of oxidative damage in mammals. At the same time, free radicals can also cause DNA strand breaks and lipid peroxidation, which in turn induces the production of peroxide MDA, so its amount also reflects the degree of free radical attack and SOD activity the body is exposed to. The size reflects the body’s ability to scavenge reactive oxygen radicals (ROS). Therefore, this article discusses the protective effect of PDTC on experimental rats after γ-ray ionizing radiation in rats, and observes its protective effect on oxidative damage of blood and tissues in rats caused by radiation. According to the experimental results, after 6.0Gy irradiation, the three PDTC administration groups can slightly increase the total SOD level of the liver and serum of rats, and reduce the MDA level of liver and serum, especially 60mg/kg and 90mg/kg are the most effective.

**Fig 5:** Total liver SOD activity after irradiation.

**Fig 6:** Total SOD activity in serum after irradiation.

## Conclusions

In this study, the NF-kB inhibitors PDTC were used to study the osteolysis process of osteoclasts induced by PDTC through a series of animal experiments. The photos after immunohistochemical staining were analyzed, the skull specimens were scanned, and the data were reconstructed by professional software. PDTC is an antioxidant and a specific inhibitor of NF-kB. PDTC inhibited the activity of NF-KB signaling pathway and promote BMP-2, OCN expression, and accelerate the formation and calcification of new bone in anterior palatal suture. PDTC can inhibit the proliferation of liver tumor cells by inhibiting the activity of NF-kB.

RETRACTED

## References

[1] GrünheidThorsten, LarsonC E, LarsonB E. Midpalatal suture density ratio: A novel predictor of skeletal response to rapid maxillary expansion, American Journal of Orthodontics and Dentofacial Orthopedics, 2017, 151(2):267–276. doi: 10.1016/j.ajodo.2016.06.043 28153155

[2] YeC, JianfengS, ZeyuanZ. Effects of lactoferrin on bone resorption of midpalatal suture during rapid expansion in rats,American Journal of Orthodontics & Dentofacial Orthopedics, 2018, 154(1):115–127. doi: 10.1016/j.ajodo.2017.09.020 29957309

[3] GarrecP, Vi-FaneB, JordanL. Rapid Maxillary Expansion (RME) Is it always matter of age?, Revue Dorthopédie Dento Faciale, 2017, 51(4):531–539. doi: 10.1051/odf/2017036

[4] RosaC B, HabibF A L, Telma Martins deAraújo. Laser and LED phototherapy on midpalatal suture after rapid maxilla expansion: Raman and histological analysis, Lasers Med, 2016, 32(2):1–12. doi: 10.1007/s10103-016-2108-3 27885521

[5] FerreiraFabíola Nogueira Holanda, Gondim J ONeto, MoreiraJosé Jeová Siebra. Effects of low-level laser therapy on bone regeneration of the midpalatal suture after rapid maxillary expansion, Lasers in Medical ence, 2016, 31(5):907–913. doi: 10.1007/s10103-016-1933-8 27056702

[6] MirK P B, MirA P B, MirM P B. A unique functional craniofacial suture that may normally never ossify: A cone-beam computed tomography-based report of two cases, Indian Journal of Dentistry, 2016, 7(1):48–50. doi: 10.4103/0975-962X.179375 27134455PMC4836098

[7] RomanykD L, ShimC, LiuS S. Viscoelastic response of the midpalatal suture during maxillary expansion treatment, Orthodontics & Craniofacial Research, 2016, 19(1):28–35. doi: 10.1111/ocr.12106 26412045

[8] HaghanifarS, MahmoudiS, ForoughiR. Assessment of midpalatal suture ossification using cone-beam computed tomography, Electronic Physician, 2017, 9(03):4035–4041. doi: 10.19082/4035 28461882PMC5407240

[9] BirlikM, KazanciogluH O, AydinM?. Effect of Energy Drink on Bone Formation in the Expanded Inter-Premaxillary Suture, Journal of Craniofacial Surgery, 2017, 28(1):285–289. doi: 10.1097/SCS.0000000000003244 27922952

[10] MengFanhua, ChengJing, SangPeng, et al. Effects of Bronchoalveolar Lavage with Ambroxol Hydrochloride on Treating Pulmonary Infection in Patients with Cerebral Infarction and on Serum Proinflammatory Cytokines, MDA and SOD. 2020, 2020doi: 10.1155/2020/798456533133226PMC7568773

RETRACTED

[11] Farinazzo Vitral RW, Fernandes, Letícia Chaves, Fraga M R. Midpalatal suture density ratio as a predictor of skeletal response to rapid maxillary expansion, American Journal of Orthodontics and Dentofacial Orthopedics, 2017, 152(3):294. doi: 10.1016/j.ajodo.2017.06.00828863905

[12] HideoS, WonM, Henrique PL. Miniscrew-assisted rapid palatal expander (MARPE): the quest for pure orthopedic movement, Dental Press Journal of Orthodontics, 2016, 21(4):17–23. doi: 10.1590/2177-6709.21.4.017-023.oin 27653260PMC5029312

[13] Bressane LB, JansonG, Oltramari-Navarro P VP. Long-term changes of alveolar buccal bone after rapid maxillary expansion in an adolescent patient, Journal of the World Federation of Orthodontists, 2016, 5(2):64–69. doi: 10.1016/j.ejwf.2016.05.003

[14] TongF, LiuF, LiuJ. Effects of a magnetic palatal expansion appliance with reactivation system: An animal experiment,American Journal of Orthodontics & Dentofacial Orthopedics, 2017, 151(1):132. doi: 10.1016/j.ajodo.2016.06.03028024766

[15] XiaoxiaC, JieG, LueW. Involvement of the Nonneuronal Cholinergic System in Bone Remodeling in Rat Midpalatal Suture after Rapid Maxillary Expansion, BioMed Research International,2016,(2016-7-10), 2016, 2016:8106067. doi: 10.1155/2016/810606727478838PMC4958416

[16] Lee RJ, MoonW, HongC. Effects of monocortical and bicortical mini-implant anchorage on bone-borne palatal expansion using finite element analysis, Am J Orthod Dentofacial Orthop, 2017, 151(5):887–897. doi: 10.1016/j.ajodo.2016.10.025 28457266PMC5472094

[17] Arnez M FM, Ribeiro L SN, Barretto GD. RANK/RANKL/OPG Expression in Rapid Maxillary Expansion, Braz Dent J, 2017, 28(3):296–300. doi: 10.1590/0103-6440201601116 29297549

[18] Samra DA, HadadR. Skeletal Age-related Changes of Midpalatal Suture Densities in Skeletal Maxillary Constriction Patients: CBCT Study, The journal of contemporary dental practice, 2018, 19(10):1260–1266. doi: 10.5005/jp-journals-10024-2414 30498183

[19] ClementE, Krishnaswamy NR. Skeletal and dentoalveolar changes after skeletal anchorage-assisted rapid palatal expansion in young adults: A cone beam computed tomography study, Apos Trends in Orthodontics, 2017, 7(3):113. doi: 10.4103/2321-1407.207220PMC535963428337417

[20] BendrihemR, VacherC. Radiologic anatomy of the maxillary artery in the pterygopalatine area applied to Le Fort 1 osteotomies, Surgical & Radiologic Anatomy Sra, 2016, 39(1):1–5. doi: 10.1007/s00276-016-1697-7 27192981

[21] DalessandriD, TonniI, DianiskovaS. Rapid palatal expansion vs quad-helix in orthodontic treatment of cleft lip and palate patients, Minerva Stomatologica, 2016, 65(2):97–103.https://xueshu.baidu.com/usercenter/paper/show?paperid=82414a3344d5da1100a200272d9e3940&site=xueshu_se 26822995

RETRACTED

[22] HoffmannC, FriederichsJ, von Rüden, Christian. Primary single suture anchor re-fixation of anterior cruciate ligament proximal avulsion tears leads to good functional mid-term results: a preliminary study in 12 patients, Journal of Orthopaedic Surgery & Research, 2017, 12(1):171. doi: 10.1186/s13018-017-0678-929132386PMC5683531

[23] AsscherickxK, GovaertsE, AertsJ. Maxillary changes with bone-borne surgically assisted rapid palatal expansion: A prospective study, Am J Orthod Dentofacial Orthop, 2016, 149(3):374–383. doi: 10.1016/j.ajodo.2015.08.018 26926025

